The article "Study on the Mechanism of Bu-Shen-He-Mai Granules in Improving Renal Damage of Ageing Spontaneously Hypertensive Rats by Regulating Th17 Cell/Tregs Balance" was published in 2022. Journal: Evid Based Complement Alternat Med.

# Study on the Mechanism of Bu-Shen-He-Mai Granules in Improving Renal Damage of Ageing Spontaneously Hypertensive Rats by Regulating Th17 Cell/Tregs Balance

**DOI:** 10.1155/2022/8315503

**Published:** 2022-04-23

**Authors:** Peng Zhang, Xu-Yu Song, Wen Li, Jian-Liang Wei, Yan-Jun Cui, Ying-Zi Qi, Xiu-Bao Chen, Yue-Hua Jiang, Chuan-Hua Yang

**Affiliations:** ^1^First Clinical Medical College, Shandong University of Traditional Chinese Medicine, Jinan 250014, China; ^2^Department of Cardiovascular, Affiliated Hospital of Shandong University of Traditional Chinese Medicine, Jinan 250014, China; ^3^Ultrasonic Room, Affiliated Hospital of Shandong University of Traditional Chinese Medicine, Jinan 250014, China; ^4^College of Health Management, Shandong University of Traditional Chinese Medicine, Jinan 250014, China; ^5^Geriatrics Department, Affiliated Hospital of Shandong University of Traditional Chinese Medicine, Jinan 250014, China; ^6^Central Laboratory, Affiliated Hospital of Shandong University of Traditional Chinese Medicine, Jinan 250014, China

## Abstract

**Methods:**

Blood pressure and urine biochemical indices were recorded. Renal blood flow was evaluated by renal ultrasonography. Transmission electron microscopy (TEM) and HE staining were used to assess kidney and spleen morphology. Renal fibrosis was assessed using Masson staining. Serum levels of IL-6, IL-10, and IL-17A were measured using ELISAs. The density of ROR*γ* and Foxp3 in the spleen was observed by immunofluorescence staining. The levels of Th17 cells and Tregs in blood were detected via flow cytometry. Transcriptome sequencing was performed to screen the targets of BSHM granules in hypertensive kidneys.

**Results:**

BSHM granules decreased SBP by 21.2 mm·Hg and DBP by 8.8 mm·Hg in ageing SHRs (*P* < 0.05), decreased the levels of urine mALB, *β*2-Mg, and NAG (*P* < 0.01), and improved renal blood flow and arteriosclerosis. BSHM granules increased IL-10 expression (*P* < 0.05) while decreasing IL-6 (*P* < 0.01) and IL-17A (*P* < 0.05) levels. BSHM granules improved Foxp3 density and the number of Tregs (*P* < 0.01) and reduced ROR*γ*t density and the number of Th17 cells (*P* < 0.01). Transcriptome sequencing identified 747 differentially expressed (DE) mRNAs in kidneys after BSHM treatment. GO analysis suggested that BSHM granules act through immunoregulation.

**Conclusions:**

BSHM granules attenuated hypertensive renal damage in ageing SHRs, by significantly increasing Tregs and decreasing Th17 cells.

## 1. Introduction

The latest study (PURE) showed that 22.3% of cardiovascular disease (CAD) events and deaths can be attributed to hypertension [1]. At the same time, hypertension is one of the main risk factors for the development and progression of chronic kidney disease (CKD) and end-stage renal disease (ESRD) [2] The intravascular pressure caused by long-range hypertension exceeds the self-adjustment of renal vessels leading to remodeling and wall thickening of small renal vessels, lumen stenosis, and a reduction in renal blood flow and the glomerular filtration rate, which in turn produces renal parenchyma injury [3]. Notably, recent studies have found that renal function in patients with hypertension decreased unexpectedly, requiring intensive antihypertensive therapy [4, 5].

The role of inflammation and immunity in the pathogenesis of hypertension has been widely recognized [6]. The infiltration of innate and adaptive immune cells in the kidney, vessel wall, and perivascular regions and other inflammatory processes, such as elevated cytokine release, reactive oxygen species (ROS) generation, and the expression of adhesion molecules are consistent features of hypertension [7, 8]. Several reports have provided evidence of a direct role of Ang II in the modification of T cell balance toward a more proinflammatory Th1 phenotype, as indicated by increased production of the Th1 cytokine IFN-*γ* [9, 10] and a decrease in Th2-mediated responses, including IL-4 production, in Ang II-infused rats [9]. Madhur et al. [11] verified that Ang II-induced hypertension was associated with increased Th17 cells and IL-17 production. Both *T* regulatory lymphocytes (Tregs) and their production of IL-10 show vascular protective effects and limit Ang II-mediated oxidative stress and vascular damage [12]. Ang II-induced endothelial dysfunction was exacerbated in IL-10 KO mice (IL-10^−/−^) [13]. Increased circulating levels of IL-6 and IL-21 and TGF-*β* receptor activation in CD4+ T cells were found to induce the development of Th17 cells and prevent the polarization of Tregs, which caused endothelial dysfunction and hypertension via an imbalance in Th17 cells/Tregs [14, 15]. Tacrolimus treatment reduced the number of Tregs and increased the level of IL-17, which was closely related to the hypertension caused by tacrolimus [16–18]. Valorie et al. [19] proposed that the Tregs and Th17 cell imbalance caused by tacrolimus contributes to the development of endothelial dysfunction and hypertension. Thus, regulating the Th17 cell/Tregs balance is a significant therapeutic strategy for the prevention and treatment of hypertensive renal damage.

Many scholars have tried to apply a variety of immunomodulatory drugs, such as PDTC, infliximab, and Ni-0101, to reduce blood pressure and improve vascular function to treat hypertension and ameliorate the damage to corresponding target organs. However, these immunomodulatory drugs may lead to cytokine release syndrome, allergic reactions, and an increased risk of cardiovascular events. Therefore, safety is still a serious obstacle to clinical application.

The human immune system develops during the congenital embryonic stage and gradually continues to develop and improve with age. Ageing directly affects the immune response. The immune homeostasis mechanism of the body gradually collapses after 65 years of age, and T cells are the main age-related immune cell population [20]. Ageing T cells have clear pathogenic potential in cardiovascular diseases, such as hypertension, atherosclerosis, and myocardial infarction [21], in which the imbalance of Th17 cells/Tregs plays an important role.

In traditional Chinese medicine (TCM), the kidney is considered the origin of the congenital constitution. The essence hidden in the kidney is the innate essence, also known as the “kidney yuan,” which transforms the innate qi of the human body, that is, the original power of life activities. As people age, the kidney qi becomes deficient, and the functions of the human body decrease, which causes dizziness. From the perspective of TCM, the immune system is also formed by the innate essence in the kidney. With the passage of time, immune function also declines. Therefore, we can regard kidney deficiency as the common basis for elderly individuals suffering from vertigo and abnormal immune function. Tonifying the kidney, that is, tonifying “kidney yuan,” is a common method for treatment of ageing-related hypertension and immune imbalance.

In the past few years, due to recent progress in TCM, the topic of treatment of hypertensive kidney damage with TCM has rushed to the forefront of medical treatment approaches and public health [2]. Recently, clinical research [5] demonstrated that prescriptions could inhibit the glomerular and tubular hyperplasia caused by high BP in SHRs, reduce urinary albumin and *β*2-microglobulin, and improve renal function. Our previous study confirmed that Bu-shen-he-mai (BSHM) decoction inhibits atherosclerosis by improving antioxidant and anti-inflammatory activities in ApoE-deficient mice [22]. Clinical studies [23, 24] have found that the antihypertensive regimen of basic antihypertensive drugs combined with BSHM Decoction can more effectively reduce the urinary protein/creatinine ratio in patients with hypertension than the basic regimen of chemical antihypertensive drugs alone, which suggests that BSHM decoction can improve renal damage. In the present study, we focused on the immunoregulation activity of BSHM granules to improve renal damage in ageing spontaneously hypertensive rats (SHRs).

## 2. Methods

### 2.1. Preparation of Bu-Shen-He-Mai (BSHM) Granules and Reagents

The dispensing granules of BSHM granules were purchased from TCM Pharmacy of Affiliated Hospital of Shandong University of Traditional Chinese Medicine (Jinan, China, Certificate: Luyao Zhizi z20120014).

BSHM treatment group: Rats were perfused with 2 g/kg/d BSHM granules, equivalent to 40 g/kg/d crude herbs and equivalent to 2 times the common clinical dosage. The chief botanical composition is shown in Table 1.

Sodium thiocyanate (S6281, Selleck, Shanghai, China), one of the main sources of thiocyanate anions, decreased IL-6 expression, increased IL-10 expression, and reduced the level of ROS. S6281 was injected intraperitoneally every second day (4.4 mg/kg/qod).

### 2.2. Animals

Animal welfare and experimental procedures were conducted in strict accordance with the principles of “Laboratory animal—Guide-lines for ethical review of animal welfare (GB/T 35892-2018)” (General Administration of Quality Supervision, Inspection and Quarantine of the People's Republic of China, 2018), and approved by the Faculty of Animal Ethics Committee of Affiliated Hospital of Shandong University of Traditional Chinese Medicine (Jinan, China). Eighty 18-month-old SHRs (SPF level, weighing 320–350 g) and twenty 18-month-old Wistar–Kyoto (WKY) rats were purchased from Beijing Vital River Laboratory Animal Technology Co., Ltd. (Certificate: SCXC (Jing) 2016–0006). All rats were housed in an air-conditioned room with a 12 h/12 h light/dark cycle at a temperature of 21 ± 1°C and humidity of 50 ± 5% and had access to food and water *ad libitum*. All rats were fed a standard chow diet for 8 weeks. Body weight and blood pressure were recorded every 2 weeks. SBP and DBP were detected with an ALC-NIBP noninvasive blood pressure analysis system. The measurements were repeated five times in parallel, and then, the average SBP and DBP values were recorded.

After 1 week of adaptation, 20 SHRs were randomly divided into two groups to confirm the efficacy of BSHM: the BSHM group (2 g/kg/d BSHM granules, equivalent to two times the common clinical dosage) and the SHR group. Ten WKY rats were used as the control group (*n* = 10). The WKY group and SHR group were intragastrically administered the same volume of saline.

Sixty SHRs were randomly divided into six groups to study the pharmacology of BSHM (*n* = 10): the BSHM group (2 g/kg/d BSHM), SHR group, BSHM + SR0987 group (2 g/kg/d BSHM, 7.14 mg/kg, administered in a single subcutaneous injection), BSHM + *S*6281 group (2 g/kg/d BSHM, 4.4 mg/kg, administered via an intraperitoneal injection every second day). Only SR0987 group (7.14 mg/kg, administered in a single intraperitoneal injection), and only S6281 group (4.4 mg/kg, administered via an intraperitoneal injection every second day). The SHRs in the model group and the WKY rats were intragastrically administered the same volume of saline (*n* = 10).

### 2.3. Biochemical Analysis

Rats were placed individually in plastic metabolism cages for 24 h for urine collection. The volume of the urine was recorded, and the urine samples were centrifuged at 3,000 r/min for 10 min at 4°C. The supernatant was used to determine the microalbumin (mALB), *β*-N-acetylglucosaminidase (NAG) and *β*2-microglobulin (*β*2-Mg) contents via biochemical assays.

### 2.4. Plasma Inflammatory Factors and Flow Cytometry

After anaesthesia with sodium pentobarbital (40 mg/kg, *i*.*p*.), blood was extracted from the heart and placed in tubes containing the anticoagulant ethylenediaminetetraacetic acid (EDTA), and plasma was separated via centrifugation.

The levels of interleukin-6 (IL-6 ELISA Kit, Cusabio Biotech, CSB-E04640r, Wuhan, China), interleukin-10 (IL-10 ELISA Kit, Cusabio Biotech, CSB-E04595r, Wuhan, China), and interleukin-17A (IL-17A ELISA Kit, Cusabio Biotech, CSB-E07451r, Wuhan, China) were measured using ELISAs.

Th17 cells were labeled with CD4-FITC and IL-17A-PE; Tregs were labeled with CD4-FITC, CD25-PerCP, and FoxP3-PE. A rat peripheral blood lymphocyte isolation kit (Solarbio, P8630, Beijing, China) was used to separate lymphocytes according to the manufacturer's protocol. Then, 6 *μ*L cocktail stimulation solution and 4 *μ*L GolgiStop protein inhibitor were added to the lymphocytes, and the mixture was gently mixed and incubated in the dark at 37°C for 5 h. The cell surface was stained with IL-17A monoclonal antibody (Thermo Fisher Scientific, 45-7177-82, Waltham, MA, USA) or Foxp3 monoclonal antibody (Thermo Fisher Scientific, 56-5773-82, Waltham, MA, USA), and the cells were fixed and permeabilized. Intracellular staining was performed. Th17 cells and Tregs were detected via flow cytometry.

### 2.5. Renal Ultrasonography

Renal ultrasonography was performed using a colour Doppler ultrasound diagnostic instrument (M5Vet, Mindray, China) under sodium pentobarbital (30 mg/kg, *i*.*p*.) anaesthesia. The segmental renal haemodynamics were recorded, and the blood parameters peak systolic blood flow velocity (Vp), diastolic minimum blood flow velocity (Vd), mean blood flow velocity (Vm), resistance index (RI), and pulsatility index (PI) were analysed using computer software (M5Vet).

### 2.6. Tissue Collection

Rats were sacrificed after treatment for 8 weeks. After anaesthesia with sodium pentobarbital (40 mg/kg, *i*.*p*.), blood was drawn via venepuncture and collected in tubes with EDTA as an anticoagulant, and plasma was separated via centrifugation. The spleens and kidneys were removed and placed on ice as soon as possible. The kidneys were subjected to haematoxylin-eosin (HE) staining, Masson staining, transmission electron microscopy, transcriptome sequencing, RT-qPCR, and Western blotting. The spleens were subjected to HE staining and immunofluorescence staining.

### 2.7. Transmission Electron Microscopy (TEM)

The extracted kidney tissue was immediately fixed in glutaraldehyde solution. Renal micromorphology was observed via TEM (×15000) (JEOL-1200, JEOL, Japan).

### 2.8. Masson Staining and HE Staining

Renal fibrosis was assessed via Masson staining. Dewaxed slices were soaked in Masson dye solution (Servicebio, G1006, Wuhan, China) according to the manufacturer's instructions and then observed under a microscope (Nikon Eclipse E100, Nikon, Japan), and images were acquired and analyzed (Nikon DS-U3, Nikon, Japan). Collagen fibers were stained blue, while muscle fibers, cellulose, and red blood cells were stained red. The fibrotic area (%) identified via Masson staining was analyzed using ImageJ.

The morphology of the spleen and kidneys was observed via HE staining. Dewaxed slices were stained with an HE dye solution set obtained from Servicebio (Servicebio, G1003, Wuhan, China) following the standard steps. The stained spleens and kidneys were observed under a microscope (Nikon Eclipse E100, NIKON, Japan), and images were acquired and analyzed (Nikon DS-U3, NIKON, Japan). The nuclei were stained blue, and the cytoplasm was stained red.

### 2.9. Immunofluorescence Staining

Spleen sections were immunostained following standard procedures. The sections were incubated with rabbit anti-ROR gamma T antibody (1 : 500, Bioss, bs-23110R, Beijing, China) or anti-FOXP3 rabbit pAb (1 : 1000, Servicebio, GB112325, Wuhan, China) at 4°C overnight. After washing steps, the sections were incubated with FITC-conjugated goat anti-rabbit IgG (1 : 200, Servicebio, GB22303, Wuhan, China) or Cy3-conjugated goat anti-rabbit IgG (1 : 500, Servicebio, GB21303, Wuhan, China) at room temperature for 30 min. Sections were observed under a fluorescence microscope. The positive rates of immunofluorescence staining were analyzed using ImageJ.

### 2.10. Transcriptome Sequencing

Total RNA was extracted from kidneys using a TRIzol reagent kit (Life Technologies, 15596–018, Carlsbad, USA) according to the standard protocol. Total RNA was further purified to avoid contamination. A total amount of 1 *μ*g RNA per sample was used as input material for the RNA sample preparations. Briefly, mRNA was purified from total RNA using poly-T oligo-attached magnetic beads. Fragmentation was carried out using divalent cations under elevated temperature in First Strand Synthesis Reaction Buffer (5X). First strand cDNA was synthesized using random hexamer primers and M-MuLV Reverse Transcriptase (RNase H-). Subsequently, second strand cDNA synthesis was performed using DNA Polymerase I and RNase H. Remaining overhangs were converted into blunt ends via exonuclease/polymerase activities. After adenylation of the 3′ ends of DNA fragments, adaptors with hairpin loop structures were ligated to prepare for hybridization. To preferentially select cDNA fragments 370–420 bp in length, the library fragments were purified with AMPure XP beads (Beckman Coulter, Beverly, USA). Then, PCR was performed with Phusion High-Fidelity DNA polymerase, Universal PCR primers, and Index (X) Primer. Finally, PCR products were purified (AMPure XP beads), and library quality was assessed on an Agilent Bioanalyzer 2100 system. Gene Ontology (GO) enrichment analysis of differentially expressed (DE) genes was implemented using the cluster Profiler R package, in which gene length bias was corrected. GO terms with corrected *P* values less than 0.05 were considered significantly enriched in differentially expressed genes. The genes were ranked according to the degree of differential expression in the two samples, and then, the predefined gene set was tested to determine whether the genes were enriched at the top or bottom of the list. Gene set enrichment analysis can include subtle expression changes.

### 2.11. Reverse Transcription-Quantitative Polymerase Chain Reaction (RT-qPCR)

After extraction with TRIzol reagent (Thermo Fisher Scientific, 10296010, Waltham, MA, USA) and quantification with a NanoDrop 2000°c spectrophotometer (Thermo Fisher Scientific, Waltham, MA, USA), total RNA samples were reverse-transcribed using a Reverse Transcriptase Kit (Sparkjade, AG0303-B, Qingdao, China). The relevant expression of RNAs was determined using the 2^−△△CT^ method. The fold change was normalized to that in the WKY group, and *β*-actin was used as an internal reference.

The primer (Sparkjade, Qingdao, China, China) sequences were as follows: SMAD3 (5′-TCGTCCATCCTGCCCTTCACC-3′/5′-ACTTCTCCTCCTGCCCGTTCTG-3′); NF-*κ*BP65 (5′-GCGGTTACGGGAGATGTGAAGATG-3′/5′-GAAGGTGGATGATGGCTAAGTGTAGG-3′); Stat3 (5′-AGGGCTTCTCGTTCTGGGTCTG-3′/5′-CTCCCGCTCCTTGCTGATGAAAC-3′); IL-6 (5′-ACTT CCAGCCAGTTGCCTTCTTG-3′/5′-TGGTCTGTTGTGG GTGGTATCCTC-3′); and TGF-*β*1 (5′-GACCGCAACAACGCAATCTATGAC-3′/5′-CTGGCACTGCTTCCCGAATGTC-3′).

### 2.12. Western Blotting Analysis

For validation of the transcriptome sequencing data, key proinflammatory *cytokine* genes, such as *IL-6*, *Smad3*, *Stat3*, *NF-κB*, and *TGF-β1*, were chosen for Western blot analysis.

Protein was extracted from the renal tissues in RIPA lysis buffer (Beyotime, P0038 B, Shanghai, China). Protein samples (30 *μ*g) were subjected to 12% sodium dodecyl sulfate-polyacrylamide gel electrophoresis. The blots were incubated at 4°C with gentle shaking overnight with primary antibodies (rabbit anti-TGF beta 1 polyclonal antibody, 1 : 1000, Bioss, bs-0086R, Beijing, China; rabbit anti-IL-6 polyclonal antibody, 1 : 1000, Bioss, bs-6309R, Beijing, China; STAT3 rabbit polyclonal antibody, 1 : 2000, Proteintech, 10253-2-AP, Rosemont, USA; rabbit anti-Smad3 polyclonal antibody, 1 : 1000, Bioss, bs-3484R, Beijing, China; rabbit anti-NF-KB polyclonal antibody, 1 : 1000, Bioss, bs-20159R, Beijing, China; rabbit anti-beta-actin (loading control) polyclonal antibody, 1 : 10000, Bioss, bs-0061R, Beijing, China). After washing steps, the blots were incubated with horseradish peroxidase conjugated to goat anti-rabbit IgG (1 : 20,000) at room temperature for 1 h. Then, they were visualized by incubation with Immobilon Western Chemiluminescent HRP Substrate (Merck Millipore, 1579205, Darmstadt, Germany) and exposed for 60 s using a Fluor Chem Q system. The bands were quantified using ImageJ (National Institutes of Health, Bethesda, Maryland, USA), and the density value was normalized to that of *β*-actin.

### 2.13. Statistical Analysis

Statistical analysis was performed using SPSS 26.0 software. The data are presented as the mean ± standard deviation (SD). Statistical analysis was performed with one-way ANOVA, followed by an LSD test. *P* < 0.05 was considered to indicate a significant difference.

## 3. Results

### 3.1. BSHM Attenuates Ageing-Related Spontaneous Hypertension

The data (*P* < 0.01, Figure 1(a)) confirmed that BSHM effectively increased the body weight of ageing SHRs. BSHM administration decreased systolic blood pressure (SBP) by 21.2 mm·Hg and diastolic blood pressure (DBP) by 8.8 mm·Hg in ageing spontaneously hypertensive rats (*P* < 0.05) (Figures 1(b) and 1(c)).

### 3.2. BSHM Improves Renal Blood Flow, Arteriosclerosis, and Renal Fibrosis in Ageing SHRs

SHRs had the higher urine levels of mALB, *β*2-Mg and NAG than WKY rats (*P* < 0.01). Compared with the SHR group, BSHM administration decreased the levels of urine mALB, *β*2-Mg and NAG (*P* < 0.01) (Figure 2(a)).

The renal blood flow in the SHR group was much worse than that in the WKY group, with slow renal artery blood flow and renal arteriosclerosis: Vp, Vd, Vm, RI and PI (*P* < 0.01), as measured by renal ultrasonography. BSHM enhanced the blood flow in the renal artery (Vp increased by 24% (*P* < 0.01), Vd increased by 62% (*P* < 0.05), and Vm increased by 38% (*P* < 0.01)) and improved the degree of renal arteriosclerosis (PI was reduced by 28% (*P* < 0.05), and RI was reduced by 10% (*P* < 0.05)) (Figure 2(b)).

Compensatory hypertrophy of renal tubules was observed in SHRs, but BSHM improved the morphology of kidneys (Figure 2(c)). TEM observation revealed that the mitochondria in SHR kidneys were obviously swollen, the density of cytoplasm was increased, and the nucleoplasm was condensed. BSHM effectively improved the morphology of SHR kidneys (Figure 2(d)). More collagen deposition was observed in SHR kidneys, which suggested an inclination toward renal fibrosis in SHRs (*P* < 0.01) (Figures 2(e) and 2(f)). BSHM decreased collagen deposition in the kidneys and improved renal fibrosis in ageing SHRs (*P* < 0.01) (Figures 2(e) and 2(f)).

### 3.3. BSHM Promotes the Immune Balance and Homeostasis

Disrupted spleen cell distribution was observed in SHRs, but BSHM improved the morphology of spleens (Figure 3(a)). SHRs had higher levels of plasma IL-6 and IL-17A (*P* < 0.01) and lower levels of IL-10 (*P* < 0.01) than WKY rats. BSHM significantly increased IL-10 (*P* < 0.01) and decreased IL-6 and IL-17A (IL-6 *P* < 0.01, IL-17A *P* < 0.05) levels in SHRs (Figure 3(b)).

Flow cytometry was used to determine the levels of both Th17 cells and Tregs in peripheral blood. Compared with the WKY group, the Th17 cell number was increased in the SHR group (*P* < 0.01), and that of Tregs decreased (*P* < 0.01). BSHM significantly increased the number of Tregs (*P* < 0.01) and decreased the number of Th17 lymphocytes (*P* < 0.01) (Figures 3(c) and 3(d)).

Immunofluorescence staining demonstrated that ROR*γ*t expression (to identify Th17 cells [25]) was increased and Foxp3 expression (to identify Tregs) was decreased in SHR rats, while BSHM obviously improved Foxp3 (*P* < 0.01) and reduced ROR*γ*t (*P* < 0.01) expression levels (Figures 3(e) and 3(f)).

### 3.4. The Target of BSHM Is Immune Regulation

A total of 40285274 to 45780200 clean reads were collected for libraries in the BSHM and SHR groups, respectively. In transcriptome sequencing, SHR demonstrated differential expression of 2847 mRNAs (1633 were downregulated and 1214 were upregulated) compared to WKY rats (fold change >2, *P* < 0.05, SHR *vs*. WKY), while 747 DE mRNAs were identified (418 were downregulated and 329 were upregulated) after BSHM treatment (fold change >2, *P* < 0.05, BSHM *vs*. SHR). A heatmap showing the DE mRNAs among SHRs, WKY rats, and BSHM-treated rats is presented in Figure 4(a). The top 10 up/downregulated mRNAs are summarized in Table 2. GO analysis (Figures 4(b) and 4(c)) suggested that BSHM modulated immunoregulation (GO: 0031347, regulation of defense response, *P* value: 1.32E-06, GO:0006954, inflammatory response, *P* value: 2.07E-06, GO:0098542, defense response to other organism, *P* value: 4.82E-08, GO:0045087, innate immune response, *P* value: 1.13E-07).

Thus, we focused on the Th17 cell/Tregs balance due to the potential activity of BSHM in immunoregulation in kidneys suggested by transcriptome sequencing.

## 4. S6281 Attenuates Hypertension in Ageing SHRs, While SR0987 Aggravates Hypertension

The data (*P* < 0.01, Figure 5(a)) confirmed that BSHM effectively increased the body weight of ageing SHRs. After eight weeks of treatment, BSHM administration decreased systolic blood pressure (SBP) by 29.5 mmHg and diastolic blood pressure (DBP) by 8.1 mm·Hg in ageing spontaneously hypertensive rats (*P* < 0.01) (Figures 5(b) and 5(c)). BSHM + *S*6281 administration decreased systolic blood pressure (SBP) by 15 mm·Hg and diastolic blood pressure (DBP) by 3.3 mm·Hg, while BSHM + SR0987 increased SBP by 31.2 mm·Hg and diastolic blood pressure (DBP) by 10 mm·Hg compared with the BSHM group (*P* < 0.01) (Figures 5(b) and 5(c)).

### 4.1. BSHM Improves Urine Biochemical Indices and Renal Fibrosis in Ageing SHRs, and the Effect Was Expanded When Treatment Was Combined with S6281 and Offset When Combined with SR0987

SHRs had higher urine levels of mALB, *β*2-Mg and NAG than WKY rats (*P* < 0.01), and BSHM administration decreased the levels of urine mALB, *β*2-Mg, and NAG (*P* < 0.01). Compared with the BSHM group, the urine levels of mALB, *β*2-Mg, and NAG were increased in the BSHM + SR0987 group (*P* < 0.01), but decreased in the BSHM + *S*6281 group (*P* < 0.01) (Figure 5(d)).

Shrinkage of glomerular loops, basement membrane thickening, and both atrophy and compensatory hypertrophy of renal tubules were observed in SHRs. Compared with the BSHM group, the BSHM + SR0987 group had a much worse renal morphology, while BSHM + *S*6281 improved the morphology of the kidneys (Figure 5(e)). Based on Masson staining, compared with the BSHM group, renal fibrosis in the SHR group and BSHM + SR0987 group was more severe (*P* < 0.01), and BSHM + *S*6281 obviously alleviated renal fibrosis (*P* < 0.01) (Figures 5(f) and 5(g)).

### 4.2. Immunoregulation of BSHM Was Expanded by Combined Treatment with S6281 and Offset by Combined Treatment with SR0987

HE staining suggested that the spleen cell distribution in SHRs was disordered. BSHM effectively improved the splenic cell distribution, and the effect was expanded after cotreatment with S6281 and offset after cotreatment with SR0987 (Figure 6(a)).

SR0987 increases IL-17 expression while reducing PD-1 expression. S6281 decreases IL-6 and increases IL-10 expression, reducing the level of ROS. BSHM increased IL-10 (*P* < 0.05) and decreased IL-6 (*P* < 0.01) and IL-17A (*P* < 0.05) expression in ageing SHRs. Compared with the BSHM group, both IL-6 and IL-17A levels were increased in the BSHM + SR0987 group (*P* < 0.01), but the IL-10 level was decreased (*P* < 0.01). BSHM + *S*6281 significantly increased IL-10 (*P* < 0.05) and decreased IL-6 and IL-17A (*P* < 0.01) expression (Figure 6(b)).

BSHM increased Tregs (*P* < 0.01) and decreased Th17 cells (*P* < 0.01) in ageing SHRs. Compared with the BSHM group, Th17 cells were increased (*P* < 0.01) and Tregs were decreased (*P* < 0.01) in the BSHM + SR0987 group. BSHM + *S*6281 significantly increased Tregs (*P* < 0.01) and decreased Th17 cells (*P* < 0.01) (Figures 6(c) and 6(d)).

Immunofluorescence staining demonstrated that ROR*γ*t expression was increased and Foxp3 expression was decreased in SHRs and BSHM + SR0987 rats, while BSHM + *S*6281 improved the status. BSHM improved Foxp3 (*P* < 0.01) and reduced ROR*γ*t (*P* < 0.01) expression in ageing SHRs. Compared with the BSHM group, ROR*γ*t was increased (*P* < 0.01), and Foxp3 was decreased (*P* < 0.01) in the BSHM + SR0987 group. BSHM + S6281 obviously improved Foxp3 (*P* < 0.01) and reduced ROR*γ*t (*P* < 0.01) expression (Figures 6(e) and 6(f)).

### 4.3. RT-qPCR

qPCR results showed that IL-6, STAT3, TGF-*β*1, NF-*κ*B, and SMAD3 expression levels were significantly higher in the SHR group than in the WKY group: IL-6 (43 times), STAT3 (25 times), TGF-*β*1 (21 times), NF-*κ*B (7 times), and SMAD3 (10 times). BSHM + *S*6281 significantly reduced the expression levels of these indicators close to the levels observed in the WKY group. The expression levels of these indicators were much higher in the BSHM + SR0987 group than in the BSHM group. BSHM and BSHM + *S*6281 significantly reduced the expression of these indicators. More details can be found in Figure 7(a).

### 4.4. Western Blotting Analysis

Western blot assays confirmed that BSHM and BSHM + *S*6281 decreased IL-6, SMAD3, Stat3, NF-*κ*B, and TGF-*β*1 protein expression, and SR0987 increased the expression of these proteins (Figures 7(b) and 7(c)), which was consistent with the RT-qPCR data and in line with the GO analysis of transcriptome sequencing.

## 5. Discussion

Hypertension-related renal damage is the second leading cause of ESRD, and coexistent hypertension plays a predominant role in the progression of most chronic kidney diseases [26, 27]. Currently, the mechanism of hypertensive renal damage is not fully understood. Immunoregulation, in addition to genetics and the environment, is involved in the process of hypertensive renal damage. One characteristic of the relationship between activation of the innate and adaptive immune systems that causes inflammation of the kidneys and hypertension is an increase in the infiltration of immune cells, including macrophages and T lymphocytes, in renal interstitial tissue [28]. It has been reported that depleting both B and T cells, such as with mycophenolate mofetil, protects against hypertension and renal disease in SHRs [29, 30].

Ageing directly affects the immune response. After 65 years of age, the immune homeostasis mechanism of the body gradually collapses. T cells are the main immune cell groups affected by ageing [20]. Ageing T cells have a clear role in pathogenicity in cardiovascular diseases, such as hypertension, atherosclerosis, and myocardial infarction [21].

BSHM is a TCM formula commonly used to treat ageing-related spontaneous hypertension in clinical practice, and the chief botanical components are HunagQi, HuangJing, SangJisheng, NvZhenzi, and NiuXi, which are used to tonify the kidney and replenish qi. The effect of BSHM on improving renal damage in ageing SHRs was investigated in the present study. Eight weeks of BSHM administration led to a successful decrease in SBP and DBP in ageing SHRs. Urinary mALB has been identified as an independent predictive factor of hypertension, cardiovascular complications, and other chronic renal diseases and is a reliable and sensitive indicator of early-stage renal injury [31]. *β*2-Mg, a protein with a relative molecular weight of 11,800, is mainly produced by human lymphocytes and serves as a sensitive indicator of the glomerular filtration rate and the reabsorption function of the proximal tubule that reflects renal injury [32–34]. Urinary NAG is a conventional marker used to assess renal injury [34]. BSHM significantly reduced the levels of urinary mALB, *β*-Mg, and NAG in SHRs, suggesting renoprotective properties of BSHM. BSHM improved renal artery blood flow and arterial stiffness, which are independent and robust predictors of chronic kidney and cardiovascular disease [35, 36]. Alleviation of hyperplasia and hypertrophy of vascular smooth muscle layers contributed to an increase in arterial compliance and a decrease in blood pressure. Injury to renal tubules plays an important role in the development of various renal diseases [37], thus, we mainly focused on the structure of renal tubules in this study. The structural and fibrotic improvement in kidneys after BSHM treatment was supposed to be an important pharmacological mechanism of BSHM.

IL-6 induces Th17 cell differentiation together with TGF-*β*, while inhibiting TGF-*β*-induced Treg differentiation, indicating that IL-6 is a very important factor in determining the Th17 cell/Tregs balance [38]. Tregs demonstrate a prominent antihypertensive effect due to their ability to produce the anti-inflammatory cytokine IL-10 [28] and reduce oxidative stress in blood vessels [39]. IL-10 is an anti-inflammatory factor secreted by Tregs and plays an important cardiovascular protective role in hypertension [12], while IL-17A is a proinflammatory factor secreted by Th17 cells that contributes to the maintenance of elevated blood pressure [11].

The transcription factor forkhead box P3 (Foxp3) controls the phenotype and function of Tregs [28]. ROR*γ*t is expressed in a subset of lamina propria T cells and is required for the expression of IL-17 [40]. The ratio of Foxp3 and ROR*γ*t contributes to the Th17 cell/Treg balance. BSHM significantly increased the density of Foxp3 in the spleen, circulating Tregs and IL-10 but decreased the density of ROR*γ*t in the spleen, circulating Th17 lymphocytes, IL-6, and IL-17A, indicating that BSHM inhibited the inflammatory response and ameliorated the Th17 cell/Treg balance. These data suggest that the immunoregulatory effect of BSHM plays an important role in improving renal damage in ageing SHRs.

Therefore, SR0987 (a ROR*γ*t agonist [41, 42]) and sodium thiocyanate (S6281, an IL-10 secretion agonist) were used to verify the immunoregulatory effect of BSHM. In this study, separate SR0987 or S6281 treatment aggravated or alleviated renal damage in ageing SHRs, respectively. The effects of BSHM were offset by BSHM combined with SR0987 but enhanced by BSHM combined with S6281.

BSHM significantly decreased systemic expression of IL-6, NF-*κ*B and Stat3 in SHRs and expression in SHR kidneys, which suggests that the Toll-like receptor signalling pathway screened out by transcriptome sequencing might be a target of BSHM.

Recently studies [43–45] have confirmed that TGF-*β*1 is the central mediator of progressive renal fibrosis and acts as a negative regulator of the immune response [46]. Smad3 is the main mediator of the biological effects of TGF-*β*1 and plays a role in promoting fibrosis [44, 47, 48]. Therapy targeting Smad3 may be a specific and effective treatment for renal fibrosis [48]. BSHM reduced both TGF-*β*1 and Smad3 expression, suggesting that BSHM brought greatly alleviated renal fibrosis and protected against the progression of hypertensive renal damage.

In conclusion, we demonstrated that BSHM granules attenuated hypertensive renal damage in ageing SHRs, improved renal structure and blood flow, and alleviated arteriosclerosis and fibrosis by significantly increasing Tregs and decreasing Th17 cells and the levels of their related inflammatory factors. Because this was an in vitro study, the results only provide clues to guide further clinical studies, which are required to confirm our findings.

## 6. Conclusions

BSHM attenuated hypertensive renal damage in ageing SHRs, mainly by balancing Th17/Treg lymphocytes and inhibiting the inflammatory response.

## Figures and Tables

**Figure 1:** BSHM attenuates ageing spontaneously hypertension in blood press. (a) Body weight (*n* = 10). (b) Systolic blood pressure (n = 10). (c) Diastolic blood pressure (n = 10). Notes: ^*∗∗*^*p* < 0.01 vs. WKY group; ^△^*P* < 0.05*P* vs. SHR group.

**Figure 2:** BSHM improves urine biochemistry, renal blood flow, arteriosclerosis, and renal fibrosis in ageing SHRs. (a) Urine biochemistry: urine mALB, urine *β*2-Mg, and urine NAG (*n* = 10). (b) Indicators of renal ultrasonography, Vp, Vm, Vd, RI, and PI (*n* = 3). (c) Representative pictures of HE staining (× 200), TEM (× 15000) (d) and Masson staining (× 200) (e) of kidneys. (f) The positive rates of Masson staining were analyzed by ImageJ (*n* = 3). Notes: ^*∗∗*^*P* < 0.01 vs. WKY group; ^△^*P* < 0.05 vs. SHR group; ^△△^*P* < 0.01 vs. SHR group.

**Figure 3:** BSHM improves the immunity of whole body and kidney and promotes the immune balance and homeostasis. (a) Representative pictures of HE staining (× 200) of spleens (n = 3). (b) The levels of plasma IL-6, IL-10, and IL-17A (*n* = 10). (c) Flow cytometry was used to determine the levels of both Th17 and Treg cells in peripheral blood (*n* = 10). (d) Representative pictures of flow cytometry (*n* = 3). (e) Representative pictures of immunofluorescence staining. Red area for Foxp3 and green area for ROR*γ*t (*n* = 3). (f) The positive rates of immunofluorescence staining were analyzed by ImageJ (*n* = 3). Notes: ^*∗∗*^*P* < 0.01 vs. WKY group; ^△^*P* < 0.05 vs. SHR group; ^△△^*P* < 0.01 vs. SHR group.

**Figure 4:** The target of BSHM is immune regulation. (a) Total of 40285274 to 45780200 clean reads were collected for libraries in BSHM and SHR group. A1, heatmap of WKY group vs. SHR group; A2, heatmap of BSHM group vs. SHR group. (b), (c) GO analysis.

**Figure 5:** BSHM improves BP, urine biochemical indices, and renal fibrosis in ageing SHRs, and the effect was expanded when treatment was combined with S6281 and offset when combined with SR0987. (a) Body weight (*n* = 10). (b) Systolic blood pressure (n = 10). (c) Diastolic blood pressure (n = 10). (d) Urine biochemistry: urine mALB, urine *β*2-Mg, and urine NAG (*n* = 10). (e) Representative pictures of HE staining (× 200) and Masson staining (× 200). (f) of kidneys (n = 3). (g) The positive rates of Masson staining were analyzed by ImageJ (*n* = 3). Notes: ^*∗∗*^*P* < 0.01 vs. WKY group; ^△△^*P* < 0.01 vs. SHR group; ^∇∇^*P* < 0.01 vs. BSHM group; ^●^*P* < 0.01 vs. BSHM group.

**Figure 6:** Immunoregulation of BSHM was expanded by combined treatment with S6281 and offset by combined treatment with SR0987. (a) Representative pictures of HE staining (× 200) of spleens (n = 3). (b) The levels of plasma IL-6, IL-10, and IL-17A (*n* = 10). (c) Flow cytometry used to determine the levels of both Th17 cells and Tregs in peripheral blood (n = 3). (d) Representative pictures of flow cytometry (*n* = 3). (e) Representative pictures of immunofluorescence staining. Red area for Foxp3 and green area for ROR*γ*t. (*n* = 3). (f) The positive rates of immunofluorescence staining were analyzed by ImageJ (*n* = 3). Notes: ^*∗∗*^*P* < 0.01 vs. WKY group; ^△^*P* < 0.05 vs. SHR group; ^△△^*P* < 0.01 vs. SHR group; ^∇∇^*P* < 0.01vs. BSHM group; *P* < 0.01 vs. BSHM group.

**Figure 7:** RT-qPCR and western blotting analysis. (a) mRNA level by RT-qPCR. The value of *y*-axis represents the multiple of each group and WKY group. IL-6R (multiple), STAT3 (multiple), TGF-*β* (multiple), NF-*κ*B (multiple), and SMAD3 (multiple) (*n* = 3). (b) The analysis of WB light density was analysed by ImageJ. IL-6R, STAT3, TGF-*β*, NF-*κ*B, SMAD3 (*n* = 3). (c) Representative pictures: western blot assay of IL-6R, STAT3, TGF-β, NF-κB, and SMAD3 (n = 3). Notes: ^*∗∗*^*P* < 0.01 vs. WKY group; ^△^*P* < 0.05 vs. SHR group, ^△△^*P* < 0.01 vs. SHR group; ^∇∇^*P* < 0.01 vs. BSHM group; *P* < 0.01 vs. BSHM group.

**Table 1:** Main botanical compositions of BSHM granules.

Herb	English name	Medicinal parts	Amount in application (g)
La radice di *Astragalus membranaceus* (HuangQi)	*Astragalus membranaceus*	Rhizome	30
Branchi e foglie di piante parassitarie della famiglia moraceae (SangJisheng)	Taxilli	Leaf	15
Polygonatum plants (huangjing)	*Polygonatum sibiricum*	Rhizome	15
Fruit of *Ligustrum lucidum* (NcZhenzi)	*Ligustrum lucidum*	Fruit	15
Dry roots of *Achyranthes bidentata* (NiuXi)	*Achyranthis bidentatae radix*	Rhizome	15

SR0987 (Selleck, Shanghai, China) is an ROR*γ*t agonist with an EC50 of 800 nM. SR0987 increases IL-17 expression while reducing PD-1 expression. SR0987 was administered via a single intraperitoneal injection (7.14 mg/kg).

**Table 2:** Top 10 up/downregulated mRNAs in transcriptome sequencing (n = 3, BSHM *vs*. SHR).

Gene name	Regulation	*P* values	log2FoldChange	Description
LOC100912599	Up	0.0002	5.5696	NADH dehydrogenase
Mapk8ip2	Up	0.0352	4.4850	Mitogen-activated protein kinase 8 interacting protein 2
Tex101	Up	0.0400	4.0397	Testis expressed 101
LOC103690026	Up	0.0003	3.8898	S-Adenosyl-L-methionine-dependent tRNA 4-demethylwyosine synthase-like
Nsun4	Up	0.01967	3.8131	NOP2/Sun RNA methyltransferase family member 4
LOC103694874	Up	3.8154	3.7990	Stromelysin-3
Tat	Up	0.0266	3.6292	Tyrosine aminotransferase
Pimreg	Up	0.0428	3.4619	PICALM interacting mitotic regulator
Efna3	Up	0.0490	3.3519	Ephrin A3
LOC100911225	Up	0.0456	3.2497	Fucose mutarotase-like
Derl3	Down	0.0100	−5.5691	Derlin 3
Hprt1	Down	0.0018	−5.1367	Hypoxanthine phosphoribosyltransferase 1
LOC100910021	Down	0.0194	−5.0797	Phosphatidylinositol 4,5-bisphosphate 3-kinase catalytic subunit beta isoform-like
Btnl9	Down	0.0098	−4.7328	Butyrophilin-like 9
Hemgn	Down	0.0356	−4.1434	Hemogen
LOC103692165	Down	0.0089	−3.7819	Rhotekin
Nhlrc4	Down	0.0260	−3.7758	NHL repeat containing 4
Cracr2b	Down	3.4593	−3.7475	Calcium release activated channel regulator 2B
Gstm3	Down	0.0219	−3.6136	Glutathione S-transferase mu 3
Vwa5a	Down	0.0137	−3.5798	von Willebrand factor A domain containing 5A

## Data Availability

The data used to support the findings of this study are included within the article.
